RETRACTED

# Evidences of Protective Potentials of Microdoses of Ultra-High Diluted Arsenic Trioxide in Mice Receiving Repeated Injections of Arsenic Trioxide

**DOI:** 10.1093/ecam/nen090

**Published:** 2011-02-14

**Authors:** Pathikrit Banerjee, Soumya Sundar Bhattacharyya, Surajit Pathak, Naoual Boujedaini, Philippe Belon, Anisur Rahman Khuda-Bukhsh

**Affiliations:** ^1^Department of Zoology, University of Kalyani, Kalyani-741235, India; ^2^Boiron Lab, 69110 Sainte-Foy-Les-Lyon, France

## Abstract

The present study was undertaken to examine if microdoses of ultra-high diluted arsenic trioxide (a potentized homeopathic remedy, Arsenicum Album 200C, diluted 10^−400^ times) have hepatoprotective potentials in mice subjected to repeated injections of arsenic trioxide. Arsenic intoxicated mice were divided into: (i) those receiving Arsenicum Album-200C daily, (ii) those receiving the same dose of diluted succussed alcohol (Alc 200C) and (iii) another group receiving neither drug nor succussed alcohol. Two other control groups were also maintained: one fed normal diet only and the other receiving normal diet and Alc-200C. Toxicity biomarkers like aspartate and alanine aminotransferases, glutathione reductase, catalase, succinate dehydrogenase, superoxide dismutase and reduced glutathione contents were periodically assayed keeping the observer “blinded”. Additionally, electron microscopic studies and gelatin zymography for matrix metalloproteinases of liver tissues were made at day 90 and 120. Blood glucose, hemoglobin, estradiol and testosterone contents were also studied. Compared to controls, Arsenicum Album-200C fed mice showed positive modulations of all parameters studied, thereby providing evidence of protective potentials of the homeopathic drug against chronic arsenic poisoning.

## 1. Introduction

Microdoses of highly diluted arsenic trioxide (As_2_O_3_ 10^−400^) was chosen to validate its ameliorative potential against repeated arsenic intoxication employing acceptable toxicity biomarkers including specific hepato-toxicity denoting protocols. Some of these biomarkers were chosen because they reflected degree of hepatotoxicity, directly or indirectly being influenced by the extent of toxicity caused by arsenic poisoning. Further, tissue damage and necrosis, often inflicted as a result of arsenic poisoning, largely contribute to improper liver function, that in turn, may cause hepatotoxicity. In view of this, liver function tests, which include the assay of enzymes like AST and ALT, were performed. These tests can throw light on the extent of liver malfunctioning and tissue damage in arsenic intoxicated mice. Therefore, positive modulation of these parameters, if any, achieved by the administration of the remedy, can be significant and supportive of its hepato-protective potential.

RETRACTED

Inorganic arsenic (iAs) acts as a tumor-promoting agent by inducing a rapid burst of reactive oxygen species (ROS) in mammalian cells, resulting in oxidative stress [1, 2] and carcinogenesis in man [3]. Cooperative defense systems that protect the body from free radical damage include the anti-oxidant enzymes [(superoxide dismutase (SOD), catalase (CAT) and indirectly glutathione reductase (GRD) and also GSH)] and nutrients. The study of these anti-oxidant enzymes was therefore considered very pertinent. Succinate dehydrogenase, an enzyme of the inner mitochondrial membrane is concerned with energy generation and respiration; hence is essential for cell survival. This parameter was therefore also included in this study. The hematological parameters like blood glucose, hemoglobin and hormonal studies were performed since they depict the physiological status of the body. Additionally, scanning and transmission electron microscopic analyses and gelatin zymography for analyzing expression pattern of matrix metalloproteinases (MMPs) were performed at day 90 and 120.

## 2. Materials

### 2.1. Animals

Thirty-six healthy adult Swiss albino mice (*Mus musculus*) of both sexes (30–40 g) served as materials for each series, six sacrificed at each fixation interval. All animal experiments were performed based on animal ethics guidelines of Institutional Animal Ethics Committee, University of Kalyani, under the supervision of Animal Welfare Committee.

### 2.2. Experimental Design

Mice were randomized and sub-divided into the following sub-sets.

### 2.3. Arsenic Intoxicated and Drug Fed Series

In all groups, injection (intraperitoneal) with 0.016% As_2_O_3_ solution (aqueous) at the rate of 1 mL/100 g body weight was performed at an interval of 7 days (Gr-1) and sacrificed at 7, 15, 30, 60, 90 and 120 days, respectively, for all groups.

A sub-group was fed Ars Alb-200C (Gr-2) once daily till sacrificed, which comprised the intoxicated drug fed series. Another sub-group (Gr-3) was fed Alc 200C. Potentized Ars Alb-200C was procured from Boiron Laboratory, Lyon, France, as also the placebo (Alc-200 C), prepared with 70% ethanol.

### 2.4. Control Series

A group of healthy mice was maintained on normal low protein diet (normal control—Gr -4). Another group of healthy mice were fed diluted succussed alcohol (Alc-200 C) at the same rate as that of As_2_0_3_, because the “vehicle" of the homeopathic remedy was ethyl alcohol (alcohol control Gr-5).

Another group of mice was injected 0.016% As_2_0_3_ every 7th day and fed Alc-200 C (intoxicated control) till they were sacrificed, to learn about modulated effect, if any, induced by ethyl alcohol on arsenic intoxicated mice.

RETRACTED

## 3. Methods

### 3.1. Preparation of Tissue Homogenates

Liver and spleen tissues were homogenized in phosphate buffer saline (pH 7.4) and centrifuged at 5000 g for 60 min. The supernatant was used for assay of the marker enzymes (glutathione reductase, superoxide dismutase, catalase and succinate dehydrogenase), reduced glutathione, aspartate aminotransferase, alanine aminotransferase and protein estimation.

### 3.2. Biochemical Analysis

The tissue homogenate was used for the assessment of AST and ALT [4], reduced glutathione content [5], catalase [6], SOD [7], SDH [8], GRD [9, 10] and protein [11].

### 3.3. Pathological Parameters

Blood glucose content was assayed by the GOD-POD End point Colorimetric assay kit supplied by Span Diagnostics Limited, Baroda (Code-B0112), India.

Hemoglobin content was determined by Sahli's method with the help of a hemometer (Marienfield, Germany).

Serum estradiol and testosterone content was assayed by using the appropriate diagnostic kit (EQUPAR srl, Saronno, Italy) with the aid of an ELISA Reader (ELDEX 3.8, USA) at 450 nm.

### 3.4. Electron Microscopic Studies

The detailed procedure of fixation and section cutting for scanning and transmission electron microscopy (SEM and TEM, respectively) have been described elsewhere [12].

### 3.5. Level of MMP Expression

For the study of MMP activity, hepatic tissue was homogenized with phosphate buffer saline (pH 7.4), followed by centrifugation in a cooling centrifuge (REMI, C 24, India). The supernatant was collected and subjected to gelatin zymography [12, 13].

### 3.6. Statistical Analysis and Scoring of Data

Statistical significance of the difference between experimental groups was calculated using Student's paired *t*-test [14] for two means. A *P* <  .05 was considered significant. One way ANOVA has also been performed. The observers were “blinded" if the sample belonged to “experimental" or “control" group at the time of scoring the data.

## 4. Results

### 4.1. Biochemical Parameters

Arsenic intoxication caused a significant rise in AST (*P* <  .05) (Table 1), ALT (*P* <  .05) (Table 2), AcP (Table 3) and AlkP (Table 4) activity levels in liver and spleen tissues when compared to the control group. The same was true for LPO activity (Table 5). Administration of Ars Alb-200C brought about considerable recuperation in the activities of AST (.05 < *P* <  .001), AcP, AlkP and ALT (.01 < *P* <  .001) and also of LPO. There was a palpable reduction in GSH contents of both the tissues in arsenic intoxicated mice (Table 6). These values were significantly increased (.05 < *P* <  .001) in drug fed mice. Catalase activity (Table 7) significantly declined (.05 < *P* <  .001) after arsenic trioxide treatment in both the liver and spleen tissues. However, there was a considerable increase of values in the drug fed mice (*P* <  .001) as compared to that of control. Similarly, both the tissues revealed a substantial depletion (.01 < *P* <  .001) in the activities of SDH enzyme (Table 7) after repeated arsenic trioxide intoxication. But Ars Alb-200C supplementation produced considerable repletion and the values were comparable to that of controls (both Gr-1 and Gr-3; *P* <  .001).

RETRACTED

The SOD levels (Table 8) showed a significant decline in its activity in both liver and spleen tissues after arsenic trioxide treatment. In Ars Alb-200C fed mice, there was considerable revival (*P* <  .05) and the values were comparable to that of controls. Arsenic intoxication resulted in significant decrease (.05 < *P* <  .001) of total GRD content in both liver and spleen tissues when compared with normal group. Administration of Ars Alb-200C resulted in significant increase (.05 < *P* <  .001) in total GRD content (Table 8) in both liver and spleen tissues as compared to arsenic intoxicated group.

### 4.2. Pathological Changes

#### 4.2.1. Blood Hemoglobin

The hemoglobin content was reduced in As_2_O_3_ + Alc200 C fed mice as compared to that of normal controls. In Ars Alb-200C fed mice (Table 9), an increase in hemoglobin level was obtained and the values were comparable to that of controls.

#### 4.2.2. Blood Glucose Content

In As_2_O_3_ and As_2_O_3_ + Alc 200C fed mice, an increase in blood sugar content was observed at successive fixation intervals, the increase being significant (*P* <  .001) at day 90 only. The increase in blood sugar content (Table 9) was so high that it exceeded the normal level. In Ars Alb-200C fed group, there was also an increase (*P* <  .001) in blood sugar content except at day 60, where a slight decrease in the said level was observed. Here, the increase was within the permissible limits and not as high as that of As_2_O_3_ and As_2_O_3_ + alcohol fed group.

#### 4.2.3. Serum Estradiol and Testosterone Concentration

Compared to intoxicated controls (Gr-1), a decrease in serum estradiol and testosterone levels (Table 10) was obtained in As_2_O_3_ and As_2_O_3_ + Alc200 C fed mice at day 90 and 120. Administration of Ars Alb-200C resulted in an increase in serum estradiol and testosterone levels in comparison to arsenic trioxide treated group.

### 4.3. Transmission Electron Microscopic Study

Contrary to the intact nuclear membrane observed in liver cells of normal (Figure 1(a)) mice and arsenic intoxicated (Figures 1(b)–1(d)) mice administered Ars Alb-200C (Figures 1(e)-1(f)), the nuclear membrane in liver cells of As_2_O_3_ intoxicated mice seemed to be broken. Destructive changes were prominent in the cristae of arsenic intoxicated mice. Furthermore, number of vacuoles was noticed in arsenic intoxicated mice. Cisternae of the Golgi bodies of arsenic intoxicated mice were absent. In arsenic intoxicated mice fed Ars Alb-200C, these features were less conspicuous.

RETRACTED

### 4.4. Scanning Electron Microscopic Study

The hepatocytes in normal controls are shown in Figures 2(a) and 2(b). Damaged hepatocytic cells were found in the arsenic intoxicated series (Figure 2(c)). Relatively little damaged hepatocytes were found in the intoxicated group that was fed Ars Alb-200C (Figure 2(d)).

### 4.5. Metalloproteinase Activity

At 90- and 120-day fixation intervals, in As_2_O_3_ and As_2_O_3_ + Alc 200C fed mice, only one band was expressed near 77 kDa (Figure 3) which presumably belonged to MMP family. However, in some mice, this band was near 97 kDa, presumably belonging to a different MMP member. In the drug fed series, the expression of the single band appeared to be somewhat less.

### 4.6. Statistical Analysis

Many of the differences in data revealed by Student's *t*-test have been found to be statistically significant at different levels, as shown in Tables 1–10. Similarly, results of one-way ANOVA also revealed significant differences among the different parameters studied (Tables 11–13).

## 5. Discussion

Arsenic compound is a protoplasmic poison that can bind to human sulphydryl-containing proteins with high affinity. Arsenic trioxide (As_2_O_3_), extracted from arsenic compound, is a powerful ancient medication for a variety of ailments with the principle of “using a toxic against another toxic" in traditional Chinese medicine. Strikingly, As_2_O_3_ treatment in a regime of 10 mg/day of intravenous infusion for 28–60 days is effective in patients with acute promyelocytic leukemia (APL) without viable toxicity in refractory to the all-trans retinoic acid (ATRA) and the conventional chemotherapy by inducing apoptosis of APL cells [15]. Notably, As_2_O_3_ exerts a broader anti-inflammatory activity by inhibition of nuclear factor, NF-*κ*B activation through induction of inhibitor of *κ*-B expression in the airways [16]. Low dosage of As_2_O_3_ may have a potential benefit in treating patients with asthma, especially in those with steroid-dependent and resistant asthma. Overall, existing data suggest a beneficial effect of As_2_O_3_ for the treatment of cancer and even inflammatory diseases. However, that even a non-material dose derived from dilution and succussions of As_2_O_3_ could show some beneficial effects in the present study is of considerable significance and of some practical application as well. To ascertain the exact amount of arsenic pushed inside the body and simulate a condition of chronic arsenic intoxication, mice were subjected to repeated injections of arsenic trioxide that inflicted hepatic damage and oxidative stress that was observed from a substantial increase in the activities of the hepatic enzymes, namely ALT and AST. An increase in the activity of these marker enzymes portrays possibility of tissue necrosis and loss of functional integrity of hepatocyte membrane. Reduction in the levels of ALT and AST towards the respective normal values by administration of Ars Alb-200C is an indication of the protective ability of the potentized homeopathic drug as well as its ability to repair hepatic tissue damage inflicted by As_2_O_3_. During hepatic injury, superoxide radicals are known to be generated at the site of damage, which in turn modulate activities of SOD and CAT, resulting in the loss of activity and accumulation of superoxide radical, which are responsible for damage of liver tissue. Decreased CAT activity is linked to the exhaustion of the enzyme as a result of oxidative stress caused by As_2_O_3_. SOD and CAT activities were brought down to near normal after treatment with Ars Alb-200C. This gives a positive indication regarding the protective efficacy of the potentized homeopathic drug.

RETRACTED

Reduced glutathione (GSH) constitutes the first line of defense against free radicals. It plays an important role in the regulation of cell proliferation and cellular defense [17]. Exposure of cells to arsenic trioxide leads to the depletion of GSH, which may also signify damage to the hepatic cells. Positive alterations in endogenous GSH have been encountered in the present investigation after administration of the homeopathic remedy, which is in line with the activities of other biomarkers. The availability of sufficient amount of GSH increased the detoxification of active metabolites of As_2_O_3_. Succinate dehydrogenase is a membrane-bound dehydrogenase linked to the respiratory chain and is a member of the Krebs' cycle [18]. Positive modulations encountered in the activity of this enzyme and those of SOD and CAT in the drug fed mice lends support to the protective ability of the remedy in cellular and sub-cellular environments. GSSG is reduced to GSH by glutathione reductase, which is NADPH-dependent. It plays a significant role in maintaining adequate amounts of GSH. Accordingly, the reduction of GRD results in decreasing GSH [18]. In As_2_O_3_ treated mice, the activity of GRD is markedly decreased. An increase in GRD activity highlights the hepato-protective ability of the remedy.

RETRACTED

Elevated blood glucose levels in As_2_O_3_ and As_2_O_3_ + alcohol fed mice was also considerably reduced in the drug fed series. The level of blood hemoglobin was markedly decreased in arsenic intoxicated group, but in the drug fed mice the level slightly increased. Similarly, serum estradiol and testosterone levels decreased markedly in arsenic trioxide injected mice. Testosterone, an anabolic steroid, is responsible for the development and maintenance of male secondary sex characters as well as growth promoting effects. Decreased testosterone levels in males may indicate hypothalamic or pituitary disorders or damage to the testis. Alternatively, decrease in the level of serum testosterone could also be implicated to a direct relationship with the increase in toxicity due to arsenic intoxication. A positive correlation can be drawn between increased SHA and an increase in testosterone level. Positive changes in the levels of these hormones were encountered in the drug fed mice. Eagon et al. [19] showed an increased level of estradiol in females of a rat model of hyperplasia.

An increase in the number of mitochondria, distorted nuclei and large black lipid droplets was observed in TEM study of liver tissues of arsenic treated mice. Similarly, in SEM study, damaged hepatocytes and hepatic chords were observed in arsenic intoxicated group. In the drug fed series, however, these features were less marked, which would also support the positive effects of the drug in ameliorating arsenic induced effect at the ultrastructural level. MMPs hydrolyze components of the extracellular matrices; these proteases play a central role in many biological processes. MMPs facilitate invasion and metastization of carcinoma cells [20]. MMPs are a family of Zn^2+^- and Ca^2+^-dependent endopeptidases secreted by both normal and transformed cells, and capable of degrading collagenous and non-collagenous components of extracellular matrix [21, 22]. Results of the present study revealed a high level of expression of metalloproteinases. This is in conformity with high levels of expression of metalloproteinases reported in pathological conditions such as wound healing, angiogenesis, tumor invasion, metastasis [23–26], arthritis, emphysema and apoptosis [27, 28]. In the drug fed mice, no overexpression of metalloproteinases was noticed. Therefore, the expression of MMPs or rather the lack of expression provides substantial evidence in favor of their anti-tumorigenic effects at the gene expression level.

How the ultra low doses of the potentized remedy could bring about multiple changes in both enzymatic and pathological parameters as well as many biomarkers is rather unclear at the present state of our knowledge. Incidentally, Khuda-Bukhsh [29–32] proposed a working hypothesis that one mechanism through which the potentized homeopathic drugs act could be through regulation of expression of certain relevant genes. This explanation seems plausible because all the biomarkers tested are regulated by specific genetic regulatory mechanisms, and without involvement of these regulatory mechanisms, such positive results could not have been achieved.

RETRACTED

## 6. Conclusion

The results of the present study suggests that Arsenicum Album 200C can be used as an interim relief measure, especially in high-risk arsenic contaminated areas, at least till arsenic-free drinking water or better strategies to manage this dreadful problem are available. However, this would need further clinical trial, preferably by others, to validate the ameliorative potentials for its homeopathic use in large scale in the arsenic contaminated areas.

## Figures and Tables

**Figure 1:** Representative photomicrographs under TEM of liver sections of normal (a), arsenic intoxicated (b–d) and arsenic intoxicated drug fed mice (e–f). BD, black droplet; ER, endoplasmic reticulum; NM, nuclear membrane; NU, nucleus; WD, white droplet.

**Figure 2:** Representative photomicrographs under scanning electron microscopy of liver sections of normal (a–b), arsenic intoxicated (c) and arsenic intoxicated drug fed (d) mice. (Magni- 1KX); H, hepatocyte; MD, mechanical disorder.

**Figure 3:** Gelatin zymogram of liver samples showing the expression of MMP in experimental mice at 120 days l. Lane 1, normal; lane 2, As_2_O_3_; lane 3: As_2_O_3_ + Alc-200; lane 4, As_2_O_3_ + Ars Alb-200; M, molecular weight marker.

**Table 1:** Mean activities of Aspartate amino transferase (AST) (nM/mg protein/min) in liver and spleen of different series of mice at different fixation intervals.

Fixation intervals in days	30 Days	60 Days	90 Days	120 Days
Series	Activity ± SE	Activity ± SE	Activity ± SE	Activity ± SE
Liver				
Negative control	0.014 ± 0.001	0.020 ± 0.000	0.011 ± 0.001	0.012 ± 0.001
Alcohol control	0.015 ± 0.002	0.022 ± 0.004	0.013 ± 0.000	0.013 ± 0.002
As_2_O_3_	0.03 ± 0.001	0.027 ± 0.001	0.035 ± 0.001	0.038 ± 0.002
As_2_O_3_ + Alcohol	0.033 ± 0.001	0.031 ± 0.003	0.040 ± 0.003	0.041 ± 0.000
As_2_O_3_ + Ars Alb-200C	0.026 ± 0.001**	0.032 ± 0.002	0.024 ± 0.003**	0.016 ± 0.004***

Spleen				
Negative control	0.011 ± 0.000	0.008 ± 0.001	0.016 ± 0.003	0.011 ± 0.000
Alcohol control	0.012 ± 0.001	0.005 ± 0.002	0.026 ± 0.001	0.012 ± 0.002
As_2_O_3_	0.025 ± 0.000	0.022 ± 0.001	0.031 ± 0.001	0.043 ± 0.000
As_2_O_3_ + Alcohol	0.027 ± 0.001	0.026 ± 0.001	0.033 ± 0.001	0.045 ± 0.001
As_2_O_3_ + Ars Alb-200C	0.02 ± 0.000***	0.012 ± 0.000***	0.022 ± 0.001***	0.018 ± 0.000***

SE, Standard error; **P < .01, ***P < .001, determined versus arsenic intoxicated Alcohol control.

RETRACTED

**Table 2:** Mean activities of Alanine amino transferase (ALT) (nM/mg protein/min) in liver and spleen of different series of mice at different fixation intervals.

Fixation intervals in days	30 Days	60 Days	90 Days	120 Days
Series	Activity ± SE	Activity ± SE	Activity ± SE	Activity ± SE
Liver				
Negative control	0.006 ± 0.001	0.008 ± 0.000	0.005 ± 0.004	0.005 ± 0.002
Alcohol control	0.008 ± 0.002	0.005 ± 0.001	0.006 ± 0.001	0.006 ± 0.003
As_2_O_3_	0.012 ± 0.000	0.015 ± 0.000	0.019 ± 0.001	0.020 ± 0.000
As_2_O_3_ + Alcohol	0.016 ± 0.002	0.019 ± 0.001	0.021 ± 0.000	0.025 ± 0.005
As_2_O_3_ + Ars Alb-200C	0.014 ± 0.001	0.012 ± 0.000***	0.009 ± 0.001***	0.005 ± 0.000***

Spleen				
Negative control	0.003 ± 0.000	0.005 ± 0.001	0.002 ± 0.001	0.003 ± 0.000
Alcohol control	0.007 ± 0.001	0.005 ± 0.002	0.002 ± 0.000	0.006 ± 0.001
As_2_O_3_	0.011 ± 0.001	0.015 ± 0.001	0.020 ± 0.001	0.024 ± 0.000
As_2_O_3_ + Alcohol	0.020 ± 0.002	0.020 ± 0.000	0.021 ± 0.003	0.028 ± 0.001
As_2_O_3_ + Ars Alb-200C	0.012 ± 0.002*	0.007 ± 0.001***	0.005 ± 0.002**	0.004 ± 0.000***

SE, Standard error; *P < .05, **P < .01, ***P < .001, determined versus arsenic intoxicated Alcohol control.

**Table 3:** Mean activities of Acid phosphatase (AcP) (nM/mg protein/min) in liver and spleen of different series of mice at different fixation intervals.

Fixation intervals in days	30 Days	60 Days	90 Days	120 Days
Series	Activity ± SE	Activity ± SE	Activity ± SE	Activity ± SE
Liver				
Negative control	0.041 ± 0.003	0.047 ± 0.001	0.010 ± 0.000	0.022 ± 0.011
Alcohol control	0.034 ± 0.005	0.046 ± 0.002	0.031 ± 0.003	0.035 ± 0.000
As_2_O_3_	0.076 ± 0.001	0086 ± 0.003	0.054 ± 0.003	0.066 ± 0.000
As_2_O_3_ + Alcohol	0.085 ± 0.001	0.090 ± 0.001	0.057 ± 0.003	0.079 ± 0.000
As_2_O_3_ + Ars Alb-200C	0.083 ± 0.002	0.069 ± 0.001***	0.046 ± 0.001**	0.044 ± 0.001***

Spleen				
Negative control	0.03 ± 0.001	0.021 ± 0.003	0.035 ± 0.000	0.03 ± 0.001
Alcohol control	0.036 ± 0.002	0.22 ± 0.005	0.031 ± 0.008	0.038 ± 0.002
As_2_O_3_	0.074 ± 0.001	0.077 ± 0.003	0.085 ± 0.001	0.092 ± 0.003
As_2_O_3_ + Alcohol	0.076 ± 0.002	0.086 ± 0.004	0.089 ± 0.005	0.098 ± 0.001
As_2_O_3_ + Ars Alb-200C	0.068 ± 0.001**	0.057 ± 0.002***	0.054 ± 0.005***	0.051 ± 0.003**

SE, Standard error; **P < .01, ***P < .001, determined versus intoxicated Alcohol control.

**Table 4:** Mean activities of Alkaline phosphatase (AlkP) (nM/100 mg protein/min) in liver and spleen of different series of mice at different fixation intervals.

Fixation intervals in days	30 Days	60 Days	90 Days	120 Days
Series	Activity ± SE	Activity ± SE	Activity ± SE	Activity ± SE
Liver				
Negative control	0.018 ± 0.001	0.012 ± 0.001	0.018 ± 0.001	0.018 ± 0.002
Alcohol control	0.037 ± 0.001	0.013 ± 0.002	0.024 ± 0.002	0.024 ± 0.003
As_2_O_3_	0.031 ± 0.002	0.035 ± 0.000	0.036 ± 0.002	0.042 ± 0.001
As_2_O_3_ + Alcohol	0.035 ± 0.003	0.039 ± 0.006	0.041 ± 0.001	0.046 ± 0.000
As_2_O_3_ + Ars Alb-200C	0.033 ± 0.001	0.025 ± 0.002	0.023 ± 0.000***	0.026 ± 0.001***

Spleen				
Negative control	0.025 ± 0.002	0.022 ± 0.003	0.012 ± 0.001	0.014 ± 0.001
Alcohol control	0.031 ± 0.001	0.026 ± 0.002	0.021 ± 0.001	0.021 ± 0.000
As_2_O_3_	0.030 ± 0.001	0.034 ± 0.004	0.043 ± 0.002	0.043 ± 0.002
As_2_O_3_ + Alcohol	0.037 ± 0.002	0.038 ± 0.002	0.045 ± 0.001	0.039 ± 0.003
As_2_O_3_ + Ars Alb-200C	0.034 ± 0.006	0.031 ± 0.002*	0.037 ± 0.001**	0.028 ± 0.001**

SE, Standard error; *P < .05, **P < .01, ***P < .001, determined versus intoxicated Alcohol control.

RETRACTED

**Table 5:** Mean lipid peroxidation (LPO) (nm/MDA/mg wet tissue) in liver and spleen of different series of mice at different fixation intervals.

Fixation intervals in days	30 Days	60 Days	90 Days	120 Days
Series	Activity ± SE	Activity ± SE	Activity ± SE	Activity ± SE
Liver				
Negative control	0.089 ± 0.020	0.05 ± 0.002	0.04 ± 0.001	0.044 ± 0.000
Alcohol control	0.094 ± 0.003	0.056 ± 0.005	0.094 ± 0.002	0.080 ± 0.009
As_2_O_3_	0.262 ± 0.013	0.277 ± 0.031	0.292 ± 0.025	0.372 ± 0.012
As_2_O_3_ + Alcohol	0.281 ± 0.010	0.246 ± 0.028	0.298 ± 0.003	0.416 ± 0.009
As_2_O_3_ + Ars Alb-200C	0.229 ± 0.010*	0.235 ± 0.028	0.139 ± 0.002***	0.093 ± 0.005***

Spleen				
Negative control	0.17 ± 0.002	0.105 ± 0.02	0.105 ± 0.002	0.030 ± 0.011
Alcohol control	0.185 ± 0.003	0.087 ± 0.004	0.118 ± 0.003	0.022 ± 0.005
As_2_O_3_	0.242 ± 0.041	0.272 ± 0.028	0.282 ± 0.002	0.296 ± 0.015
As_2_O_3_ + Alcohol	0.262 ± 0.040	0.278 ± 0.006	0.296 ± 0.023	0.396 ± 0.010
As_2_O_3_ + Ars Alb-200C	0.232 ± 0.034	0.239 ± 0.014*	0.165 ± 0.004**	0.109 ± 0.006***

SE, Standard error; *P < .05, **P < .01, ***P < .001.

**Table 6:** Mean reduced glutathione (GSH) (nm/mg tissue) in liver and spleen of different series of mice at different fixation intervals.

Fixation intervals in days	30 Days	60 Days	90 Days	120 Days
Series	Activity ± SE	Activity ± SE	Activity ± SE	Activity ± SE
Liver				
Negative control	0.006 ± 0.001	0.006 ± 0.002	0.007 ± 0.001	0.009 ± 0.001
Alcohol control	0.003 ± 0.001	0.003 ± 0.001	0.007 ± 0.002	0.007 ± 0.001
As_2_O_3_	0.004 ± 0.000	0.002 ± 0.001	0.001 ± 0.000	0.001 ± 0.000
As_2_O_3_ + Alcohol	0.005 ± 0.000	0.003 ± 0.001	0.002 ± 0.000	0.001 ± 0.000
As_2_O_3_ + Ars Alb-200C	0.005 ± 0.001	0.006 ± 0.000*	0.006 ± 0.000**	0.008 ± 0.000***

Spleen				
Negative control	0.005 ± 0.001	0.007 ± 0.001	0.009 ± 0.001	0.009 ± 0.002
Alcohol control	0.006 ± 0.002	0.005 ± 0.001	0.008 ± 0.001	0.008 ± 0.000
As_2_O_3_	0.004 ± 0.000	0.003 ± 0.000	0.002 ± 0.001	0.001 ± 0.000
As_2_O_3_ + Alcohol	0.004 ± 0.000	0.004 ± 0.000	0.002 ± 0.000	0.002 ± 0.000
As_2_O_3_ + Ars Alb-200C	0.004 ± 0.000	0.006 ± 0.001	0.007 ± 0.001**	0.008 ± 0.001***

SE, Standard error; *P < .05, **P < .01, ***P < .001, determined versus intoxicated Alcohol control.

RETRACTED

**Table 7:** Catalase and Succinate dehydrogenase activities in liver and spleen of different series of mice at 90 and 120 days fixation interval.

Table-1	Succinate dehydrogenase (*μ*mol/mg protein)				Catalase (unit enzyme/mg protein)			
Series	90 days		120 days		90 days		120 days	
	Liver	Spleen	Liver	Spleen	Liver	Spleen	Liver	Spleen
Negative control	530.00 ± 1.58	487.00 ± 0.32	550.00 ± 1.26	500.00 ± 0.63	8.80 ± 0.003	5.50 ± 0.00	8.70 ± .001	8.20 ± 0.002
Alcohol control	541.00 ± 1.26	488.00 ± 0.63	557.00 ± 0.63	498.00 ± 0.95	8.60 ± 0.001	5.30 ± 0.01	8.50 ± 0.001	8.40 ± 0.001
As_2_O_3_	283.00 ± 1.90	272.00 ± 1.59	262.00 ± 0.63	261.00 ± 1.26	4.36 ± 0.005	2.30 ± 0.02	2.95 ± 0.003	1.86 ± 0.002
As_2_O_3_ + Alcohol	270.00 ± 0.63	256.00 ± 0.95	268.00 ± 0.95	230.00 ± 1.30	3.11 ± 0.002	1.90 ± 0.01	2.50 ± 0.01	1.40 ± 0.001
As_2_O_3_ + Ars Alb-200C	495.00 ± 0.013***	428.00 ± 0.01***	512.00 ± 0.33***	453.00 ± 1.38***	6.1 ± 0.001***	5.29 ± 0.003***	6.69 ± 0.002***	6.21 ± 0.002***

SE, Standard error; ***P < .001, determined versus intoxicated Alcohol control.

**Table 8:** Glutathione reductase (*μ*mol/mg protein/min) and Superoxide dismutase (unit enzyme/mg protein) in liver and spleen of different series of mice at 90 and 120 days fixation interval.

Table-1	Glutathione reductase (*μ*mol/mg protein/min)				Superoxide dismutase (unit enzyme/mg protein)			
Series	90 days		120 days		90 days		120 days	
	Liver	Spleen	Liver	Spleen	Liver	Spleen	Liver	Spleen
Control	24 ± 0.010	20 ± 0.201	23.63 ± 0.010	20.85 ± 0.010	0.052 ± 0.031	0.050 ± 0.010	0.049 ± 0.010	0.051 ± 0.007
Alcohol control	21 ± 0.020	22 ± 0.110	22 ± 0.010	22 ± 1.30	0.056 ± 0.011	0.051 ± 0.012	0.051 ± 0.007	0.048 ± 0.010
As_2_O_3_	9.2 ± 0.122	10 ± 0.211	8 ± 0.158	8.9 ± 0.066	0.011 ± 0.006	0.015 ± 0.002	0.010 ± 0.001	0.012 ± 0.131
As_2_O_3_ + Alcohol	10 ± 0.447	12 ± 0.103	9 ± 0.224	11 ± 1.33	0.014 ± 0.010	0.013 ± 0.007	0.009 ± 0.003	0.010 ± 0.004
As_2_O_3_ + Ars Alb-200C	19 ± 0.316***	16 ± 0.010***	22 ± 0.158***	18.6 ± 1**	0.037 ± 0.012	0.031 ± 0.010	0.061 ± 0.008***	0.052 ± 0.007**

SE, Standard error; **P < .01, ***P < .001, determined versus intoxicated Alcohol control.

RETRACTED

**Table 9:** Mean hemoglobin and Mean Blood sugar (mg/dl) content in different series of mice at different fixation intervals.

Fixation intervals in days	30 Days	60 Days	90 Days	120 Days
Series	Activity ± SE	Activity ± SE	Activity ± SE	Activity ± SE
Mean hemoglobin				
Negative control	14.1 ± 0.006	13.8 ± 0.007	16.6 ± 0.410	17.1 ± 0.170
Alcohol control	14.0 ± 0.009	14.6 ± 0.019	15.9 ± 0.039	17.0 ± 0.190
As_2_O_3_	12.8 ± 0.008	11.9 ± 0.004	11.2 ± 0.710	10.17 ± 0.190
As_2_O_3_ + Alcohol	11.6 ± 0.012	11.1 ± 0.004	10.7 ± 0.470	10.14 ± 1.490
As_2_O_3_ + Ars Alb-200C	14.0 ± 0.007***	12.7 ± 0.014***	15.17 ± 0.750***	16 ± 0.710**

Mean Blood sugar				
Negative control	84.731 ± 0.082	82.156 ± 0.054	85.76 ± 0.970	82.240 ± 0.840
Alcohol control	86.426 ± 0.056	84.286 ± 0.076	90.84 ± 1.760	80.740 ± 1.460
As_2_O_3_	111.743 ± 0.121	109.410 ± 0.238	162.45 ± 2.470	175.080 ± 2.890
As_2_O_3_ + Alcohol	117.412 ± 0.185	121.146 ± 0.089	180.48 ± 1.850	182.790 ± 1.050
As_2_O_3_ + Ars Alb-200C	104.131 ± 0.120***	97.420 ± 0.423***	99.78 ± 0.240***	92.460 ± 1.080***

SE, Standard error; **P < .01, ***P < .001, determined versus intoxicated Alcohol control.

**Table 10:** Mean Serum testosterone (ng/mL) and Mean Serum Estradiol (pg/ml) levels in different series of mice at different fixation intervals.

Fixation intervals in days	90 Days	120 Days
Series	Activity ± SE	Activity ± SE
Mean Serum testosterone		
Negative control	5.10 ± 0.160	5.40 ± 0.030
Alcohol control	5.60 ± 0.130	5.50 ± 0.040
As_2_O_3_	0.98 ± 0.010	1.21 ± 0.020
As_2_O_3_ + Alcohol	2.54 ± 0.020	2.68 ± 0.010
As_2_O_3_ + Ars Alb-200C	1.87 ± 0.020***	1.43 ± 0.015***

Mean Serum Estradiol		
Negative control	42.00 ± 1.900	46.00 ± 1.260
Alcohol control	48.00 ± 0.840	51.00 ± 1.580
As_2_O_3_	33.00 ± 0.630	32.00 ± 0.710
As_2_O_3_ + Alcohol	31.00 ± 1.260	28.00 ± 1.210
As_2_O_3_ + Ars Alb-200C	39.00 ± 1.260**	48.0 ± 0.840***

SE, Standard error; **P < .01, ***P < .001, determined versus intoxicated Alcohol control.

**Table 11:** One way ANOVA for different hepatic enzymes.

Source of	AST			ALT			LPO			GSH			Catalase			SDH			SOD		
variation	df	F	Sig.	df	F	Sig.	df	F	Sig.	df	F	Sig.	df	F	Sig.	df	F	Sig.	df	F	Sig.
Between groups	23	14.72	0.000*	23	35.93	0.000*	23	990.89	0.000*	23	2.51	0.001*	23	54.52	0.000*	23	172.80	0.000*	23	2.62	0.000*
Within groups	72			72			72			72			72			72			72		

*P < .05.

**Table 12:** One way ANOVA of different spleen enzymes.

Source of variation	AST activity			ALT activity			GSH activity			CAT activity			SDH activity			SOD activity		
	df	F	Sig.	df	F	Sig.	df	F	Sig.	df	F	Sig.	df	F	Sig.	df	F	Sig.
Between groups	23	39.131	0.000*	23	30.120	0.000*	23	3.160	0.000*	23	100.361	0.000*	23	91.231	0.000*	23	3.002	0.000*
Within groups	72			72			72			72			72			72		

*P < .05.

RETRACTED

**Table 13:** One way ANOVA of blood parameters.

Source of Variation	Blood Hb			Blood Sugar			Serum Testosterone			Serum Estadiol		
	df	F	Sig.	df	F	Sig.	df	F	Sig.	df	F	Sig.
Between groups	23	63.268	0.000*	23	750.120	0.000*	23	28.160	0.000*	23	20.361	0.000*
Within groups	72			72			72			72		

*P < .05.
